This article has been retracted.

# Human Schlafen 5 Inhibits Proliferation and Promotes Apoptosis in Lung Adenocarcinoma via the PTEN/PI3K/AKT/mTOR Pathway

**DOI:** 10.1155/2021/6628682

**Published:** 2021-03-23

**Authors:** Xuefeng Gu, Li Zhou, Lei Chen, Huiqing Pan, Rui Zhao, Weiwei Guang, Guoqing Wan, Peng Zhang, Dingsheng Liu, Li-Li Deng, Weiming Zhao, Changlian Lu

**Affiliations:** ^1^Shanghai University of Medicine & Health Science Affiliated Zhoupu Hospital, Shanghai, China; ^2^Shanghai Key Laboratory of Molecular Imaging, Shanghai University of Medicine & Health Sciences, Shanghai, China; ^3^Shanghai University of Traditional Chinese Medicine, Shanghai, China; ^4^Department of Oncology, The Second Affiliated Hospital of Harbin Medical University, Harbin, Heilongjiang, China; ^5^Qiqihar Medical University, Qiqihar, Heilongjiang, China

## Abstract

**Background:**

Human Schlafen 5 (SLFN5) is reported to inhibit or promote the proliferation of several specific types of cancer cells by our lab and other researchers. We are curious about its implications in lung adenocarcinoma (LUAC), a malignant tumor with a high incidence rate and high mortality.

**Method:**

Lentiviral stable transfections of SLFN5-specific shRNA for knockdown and SLFN5 full-length coding sequence for overexpression were performed in LUAC cell for proliferation analysis in vitro and in vivo in nude mice. Clinical LUAC samples were collected for immunohistochemical analysis of SLFN5 protein levels.

**Results:**

We found that knockdown of endogenous SLFN5 upregulates cancer cell proliferation while inhibiting apoptosis. Besides, SLFN5 inhibition on proliferation was also observed in a nude mouse xenograft model. In contrast, overexpression of exogenous SLFN5 inhibited cell proliferation *in vitro* and *in vivo* and promoted apoptosis. As to the signaling pathway, we found phosphatase and tensin homolog on chromosome 10 (PTEN) was positively regulated by SLFN5, while its downstream signaling pathway AKT/mammalian target of rapamycin (mTOR) was inhibited. Moreover, compared with adjacent normal tissues, SLFN5 protein levels were markedly decreased in lung adenocarcinoma tissues. In conclusion, these suggest that human SLFN5 plays inhibitory roles in LUAC progression through the PTEN/PI3K/AKT/mTOR pathway, providing a potential target for developing drugs for lung cancer therapy in the future.

## 1. Introduction

Increasing evidence has shown that the Schlafen family (SLFN for human/Slfn for mouse) functions in both the immune system and malignant tumors [1–10]. The Schlafen family was firstly reported to play regulatory roles in thymocyte maturation and activation in mice in 1998 [1] and was subsequently found to be conservative between mice and humans [2–5]. Of the 11 mouse Slfn members, Slfn1 and 8 inhibit T cell growth [5], Slfn2 and 3 inhibit proliferation and/or anchorage-independent growth of mouse malignant melanoma and renal cell carcinoma cells [11], and Slfn5 exhibits antineoplastic effects in mouse renal cell carcinoma cells. Of the human SLFN members, SLFN1 promotes cell cycle arrest through cyclin D1 inhibition in NIH3T3 cells [12]. Generally, some members of the human and mouse SLFN/Slfn families exert inhibitory roles in the proliferation of T cells and several specific carcinoma cell types.

However, with respect to the role of human SLFN5 in cancer cell proliferation, the reports are conflicting. Firstly, knockdown of SLFN5 promotes soft agar colony formation/anchorage-independent growth of human melanoma cells [8], but it did not affect the proliferation of renal cell carcinoma (RCC) cells [9] and even promoted glioblastoma cell growth [13]. Secondly, SLFN5 expression correlates with better overall survival in a large cohort of patients with RCC [9]. In contrast, it correlates with poor overall survival in patients suffering from glioblastoma [13]. These contradictory results in different types of cancers prompted us to investigate SLFN5 functions in other malignant cancers, particularly lung cancer, one of the most malignant tumors [14, 15]. In our recent report, we found that SLFN5 suppresses cancer cell migration and invasion by inhibiting MT1-MMP expression via the *β*-catenin pathway [16] and that SLFN5 can affect the epithelial morphology of breast cancer cells by downregulating the transcription of ZEB1 [17]. However, whether SLFN5 plays regulatory roles in lung cancer cell proliferation and apoptosis is not yet known.

Phosphatase and tensin homolog on chromosome 10 (PTEN) is a potent tumor suppressor gene that relies on its lipid phosphatase activity to catalyze the conversion of phosphatidylinositol-3,4,5-triphosphate (PIP3) to PIP2 by dephosphorylating the 3-position of the inositol ring of PIP3, thereby antagonizing phosphoinositide-3-kinase (PI3K) signaling and repressing multiple cellular processes, including cell cycle progression, proliferation, survival, motility, and metastasis [18–22]. PTEN is deficient or downregulated in several cancers, such as endometrial carcinoma [23], glioblastoma multiforme [24, 25], skin cancer [26], breast cancer [27], prostate cancer [28], and lung cancer [29]; therefore, elevated levels of PIP3 promote cellular growth and proliferation while suppressing apoptosis [23–30]. In lung cancer, PTEN is regulated by p53 [31, 32], Oct4 [33], c-Jun [34], and NF-kappa B [35]. Epigenetic silencing by both gene promoter methylation and histone modification suppresses PTEN expression [36, 37]. Loss of PTEN expression is observed in the majority of lung cancers; however, the mechanism by which PTEN expression is regulated in lung cancer has not been fully elucidated.

In the present study, we observed that SLFN5 protein levels were significantly reduced in lung adenocarcinoma compared with adjacent normal tissues. Knockdown of SLFN5 promoted lung cancer cell proliferation and inhibited apoptosis, and vice versa. We also found that SLFN5 exerts these effects through regulating PTEN/PI3K/AKT/mTOR pathways. This is the first report that human SLFN5 exerts inhibitory roles in lung cancer with respect to cell tumorigenesis and progression, providing a potential target for developing novel drugs for lung cancer therapy in the future.

## 2. Materials and Methods

### 2.1. Cell Culture

The human lung adenocarcinoma cell line A549 from American Type Culture Collection (ATCC; Manassas, VA, USA) was cultured in high glucose Dulbecco's modified Eagle's medium (DMEM; Gibco, NY, USA) supplemented with 10% fetal bovine serum (FBS; Gibco), 100 U/ml penicillin, and 100 mg/ml streptomycin and maintained at 37°C in 5% CO_2_.

### 2.2. Construction of Lentiviral Vectors of SLFN5 shRNA and Overexpression Recombinant

To obtain SLFN5 shRNA plasmid, the targeting sequences specific for SLFN5 (5′-GACUCAGACUCCAACGAAUTT-3′) were constructed into a lentiviral vector and a scrambled shRNA lentiviral vector was constructed as a negative control. SLFN5 coding sequence (NM_144975.3) was amplified using PCR and ligated into a lentiviral vector. The lentiviral vectors contain eGFP expression elements facilitating for monitoring positive cells under fluorescence microscopy. Prepared lentiviral particles were transfected into A549 cells, and puromycin was used to selected positive cells. Real-time PCR and Western blotting were used to confirm SLFN5 knockdown and overexpression efficiencies.

### 2.3. Western Blot

Western blot was performed routinely, and antibodies were used as follows. PTEN (D4.3) mAb (Cat # 9188S), Phospho-AKT (S473) (D9E) mAb (Cat # 4060S), TCF1/TCF7 (C63D9) mAb (Cat # 2203S), Phospho-mTOR (Ser2448) (D9C2) mAb (Cat # 5536T), mTOR (7C10) mAb (Cat # 2983T), Phospho-GSK-3-beta (S9) (D85E12) mAb (Cat # 5558S), *β*-catenin (D10A8) mAb (Cat #8480), caspase-3 (8G10) mAb (Cat #9665), cleaved caspase-3 (Asp175) (5A1E) mAb (Cat #9664), Bax (D2E11) mAb (Cat #5023), cyclin D1 antibody (Cat #2922), and actin antibody are all from Cell Signaling Technology. SLFN5 antibody (Cat #HAP017760) was from Sigma-Aldrich. The secondary antibodies, anti-rabbit or anti-mouse, were obtained from Beyotime (Shanghai, China). Membranes were reacted with enhanced chemiluminescence lighting reagent (ECL; Amersham Pharmacia, NJ, USA) and exposed to X-film in the dark.

### 2.4. Quantitative Real-Time PCR

Cells were lysed with Trizol reagent (Invitrogen, CA, USA), and total RNA was isolated and reverse-transcribed into cDNA using the Superscript First-Strand Synthesis System (Invitrogen, CA, USA) with random primers. Quantitative real-time PCR was performed using the SYBR Green Master Mix (Applied Biosystems, USA) to analyze gene expression with *β*-actin as an internal control. Primers used were SLFN5, forward 5′-CATCCGACGCATCACCGATCTG-3′ and reverse 5′-CATCCGACGCATCACCGATCTG-3′; PTEN, forward 5′-TTGTGGTCTGCCAGCTAAA-3′ and reverse 5′-CGCTCTATACTGCAAATGCT-3′; and *β*-actin, forward 5′-TACCTCATGAAGATCCTCACC and reverse 5′-TTTCGTGGATGCCACAGGAC-3′ [38].

### 2.5. Immunofluorescence Assay

Cells were cultured in cover glass chambers and fixed in 1% paraformaldehyde for 5 min and permeabilized with 1‰ Triton X-100 for 3 min. Cells were treated with 3% goat serum for 30 min at room temperature and incubated with SLFN5 antibody (1 : 100), or Ki-67 antibody (1 : 100) overnight. Cells were then incubated with Alexa Fluor594-labelled secondary antibodies (1 : 1000) (Invitrogen, USA) for 1 hour at room temperature in darkness. Nuclei were counterstained with DAPI, and fluorescent images were captured using confocal fluorescence microscopy (Leica; Germany).

### 2.6. Cell Counting Kit-8 Test for Proliferation Assay

For cell proliferation assay, 2000 cells in 100 *μ*l cultural medium were added to a well of 96-well plates and 10 *μ*l of Cell Counting Kit-8 (CCK-8) solution was added to each well. After incubation for 1 hour in a 37°C cell incubator, the absorbance of product formazan was determined at 450 nm. Experiments were performed at least 3 times, and data were analyzed as mean ± S.D.

### 2.7. Terminal Deoxynucleotidyl Transferase-Mediated Nick-End Labeling (TUNEL) Detection

Cell samples were fixed with 4% paraformaldehyde and permeabilized with 1‰ Triton X-100. After 3 washes with PBS, samples were added with 50 *μ*l of TUNEL solution followed by incubation in the dark for 1 hr at 37°C. DAPI was used to counterstain nuclei. Fluorescence images were captured using fluorescence microscopy, TUNEL-positive products presenting red fluorescence. Experiments were performed at least 3 times, and data were analyzed as mean ± S.D.

### 2.8. Flow Cytometry Determination of Apoptosis

Annexin V labeled with 647 nm fluorescent was used to detect apoptosis of phosphatidylserine on the surface of the cell membrane using flow cytometry. Cells were digested with an appropriate amount of pancreatic enzyme, and the cell lysates were collected for apoptosis assay. Cells were gently resuspended with 200 *μ*l of Annexin V labeled with 647 nm fluorescent and incubated with 10 *μ*l of propidium iodide dye solution at room temperature avoiding light and then placed on ice for flow cytometry detection (Annexin V, 647 nm fluorescence, and propidium iodide, red fluorescence). Apoptosis cell percentages were calculated and analyzed as mean ± S.D. (*n* = 3).

### 2.9. Plate Colony Formation Assay

Cultured cells in the logarithmic growth stage were digested with 0.25% trypsin and blown into single cells. A total of 1000 cells in a 2 ml culture medium were put in a well of 6-well plates and dispersed evenly. A single cell grew into a colony during a 2- or 3-week cultural period, and colonies over 10 cells were counted under a microscope and analyzed as mean ± S.D. (*n* = 3).

### 2.10. Nude Mouse Xenograft Model

SLFN5 knockdown or shRNA control cells (2 × 10^6^ cells per mouse) were mixed with BD Matrigel in a 1 : 1 ratio and injected subcutaneously into the left axilla of 6-week-old male nude mice (*n* = 9). For SLFN5 overexpression and Vector control cell inoculation, 1 × 10^7^ cells were used per mouse. Tumor sizes, with the longest diameter for length, the shortest diameter for width, were measured every 5 days, and the sizes and volumes were determined through external measurements and calculated by the formula: *V* = [*L* × *W*^2^] × 0.52 (*V* = volume, *L* = length, and *W* = width) [39]. When the largest tumor grew to 1.5 cm in length, the mice were sacrificed for tumor separation.

### 2.11. Lung Adenocarcinoma Histochemistry Analysis

The collection and treatment of tissue samples from lung adenocarcinoma patients met the requirements of the ethics committee of Shanghai University of Medical and Health Sciences. The samples were fixed with 10% paraformaldehyde, dehydrated with xylene gradient, embedded in paraffin, and sliced to a thickness of 4 *μ*m. Slides were incubated with anti-SLFN5 antibody, or anti-PTEN, at 1 : 100 dilution for 2 hr followed by secondary antibody incubation and reaction with DAB peroxidase substrate. Slides were also stained with H&E routinely. The staining results were read and given the results back to back by two experienced pathologists.

## 3. Results

### 3.1. Knockdown of SLFN5 Promotes and Overexpression of SLFN5 Suppresses A549 Cell Proliferation

SLFN5 is reported to exert differential effects on the proliferation of distinct cancer cell types. It inhibits melanoma cell proliferation but has no effect on renal cell carcinoma cell proliferation, while promoting glioblastoma growth. The lung adenocarcinoma cell line A549, the most commonly used cell line in the lung cancer studies, exhibits moderate expression levels of SLFN5 and was therefore adopted for both knockdown and overexpression assays in the present study. We constructed SLFN5 stable knockdown cell lines using SLFN5-specific shRNA (ShSLFN5) and scrambled shRNA as a control (ShCtrl). Meanwhile, SLFN5 overexpressing cell lines were created with a lentiviral SLFN5 recombinant vector (SLFN5) and empty vector as a control (Vector). Knockdown and overexpression efficiencies were confirmed as shown in Figure 1(a). Immunostaining of SLFN5 showed its localization to the nucleus (Figure 1(b)). During the 5- to 7-day culture periods, the numbers of ShSLFN5 cells were significantly greater than ShCtrl cells, while the numbers of SLFN5 cells were significantly less than Vector cells (Figure 1(c)). Moreover, proliferation was determined by the production of formazan using the CCK-8 detection kit. ShSLFN5 cells produced increased formazan compared to ShCtrl cells, while SLFN5 cells produced reduced formazan compared to Vector cells (Figure 1(d)). Ki-67, a nonhistone nucleoprotein that is commonly expressed in proliferation G1, S, G2, and mitotic phases, but not in G0 resting phase [40], was assessed by immunofluorescence staining. Ki-67-positive cells were present at higher percentages in the ShSLFN5 group compared to the ShCtrl group, while Ki-67-positive cells were significantly decreased in SLFN5 cells relative to Vector cells (Figure 1(e)). SLFN5's inhibitory effect on A549 cell proliferation was further confirmed by colony formation assays, with significantly more colonies observed in ShSLFN5 cells than in ShCtrl cells and evident decreases in SLFN5 cells compared to Vector cells (Figure 1(f)). Cyclin D1, a positive regulator of the G1/S phase of cell cycle and proliferation, is regarded as a biomarker of cancer progression [41], and its levels were enhanced in ShSLFN5 cells compared to ShCtrl cells and were suppressed in SLFN5 cells relative to Vector cells (Figure 1(g)). These findings demonstrate that SLFN5 inhibits A549 proliferation.

### 3.2. Knockdown of SLFN5 Suppresses and Overexpression of SLFN5 Promotes Apoptosis of A549 Cells

Whether the SLFN family is related to the apoptosis pathway has not been previously reported. To evaluate the relationship of SLFN5 with apoptosis, flow cytometry analyses of apoptosis were performed. In ShSLFN5-A549-transfected cells, both early and late apoptotic percentages were lower than in ShCtrl-A549 cells, and total apoptotic percentages decreased (Figure 2(a)). In contrast, overexpression of SLFN5 enhanced apoptotic cell percentages of both early and late apoptosis, and total apoptosis was increased compared with Vector-transfected A549 cells (Figure 2(b)), indicating that SLFN5 promotes apoptosis in A549 cells. To further verify the role of SLFN5 in apoptosis, TUNEL fluorescence staining was performed to detect fragmental DNA. TUNEL staining was almost undetectable in ShSLFN5-transfected cells (Figure 2(c)). In contrast, the numbers of positively stained cells were significantly increased in SLFN5 overexpression cells (Figure 2(d)). Bax, a member of the bcl-2 family, promotes mitochondrial apoptotic processes by binding to the mitochondrial membrane and releasing cytochrome C into the cytosol to trigger apoptosis [42]. Bax levels were decreased in ShSLFN5-transfected cells compared to ShCtrl cells. Meanwhile, Bax was increased in SLFN5-transfected cells compared to Vector cells. Caspase-3, a critical executioner of apoptosis, requires proteolytic processing of zymogen into activated cleaved caspase-3, responsible for the proteolytic cleavage of many key proteins [43]. Cleaved caspase-3 was decreased in ShSLFN5-transfected cells compared to ShCtrl cells but was increased in SLFN5 cells compared to Vector cells (Figures 2(e) and 2(f)). Together, these results indicate that SLFN5 promotes apoptosis in A549 cancer cells.

### 3.3. Knockdown of SLFN5 Promotes but Overexpression of SLFN5 Inhibits A549 Cell Growth in Nude Mice

The above proliferation and apoptosis results were obtained from *in vitro* cell culture; however, under the much more complex *in vivo* environment, rich in multiple regulatory cytokines and growth factors, various matrices, infiltrated cells, and vascular tissues, the functions of SLFN5 are largely unknown. To determine the effects of SLFN5 on tumor growth *in vivo*, A549 lung adenocarcinoma cells with SLFN5 knockdown or overexpression were subcutaneously injected into male nude mouse axilla regions. Over approximately 30 days, tumors growing from A549 cells transfected with ShSLFN5 grew significantly larger than those from ShCtrl-transfected cells, both with respect to tumor volume and weight (Figures 3(a)–3(d)). Meanwhile, tumors from SLFN5-transfected cells were markedly smaller, both in volume and weight, than those from Vector-transfected cells (Figures 3(e)–3(h)). This *in vivo* tumor growth data was entirely consistent with the *in vitro* cell culture results, indicating that SLFN5 plays inhibitory roles in lung cancer cells during tumorigenesis.

### 3.4. SLFN5 Regulates the p-AKT/mTOR Pathway via Transcriptional Regulation of PTEN mRNA

In our previous study, we found that stabilized dephosphorylated *β*-catenin translocates into the nucleus in SLFN5-siRNA-treated breast cancer MCF7 cell lines [16], so we primarily examined GSK-3*β*/*β*-catenin and its up- and downstream signaling molecules in A549 cells, observing that the GSK-3*β*/*β*-catenin pathway was regulated in response to SLFN5 in A549 cells, i.e., activated by SLFN5 knockdown, and was blocked in response to SLFN5 overexpression (Figure 4(a)). These findings support the conclusion that SLFN5 regulates cyclin D1 expression and proliferation (Figure 1). GSK-3*β* upstream molecule, such as pAKT, which is involved in cell survival, was activated in response to SLFN5 knockdown, and vice versa. mTOR protein, activated by the PI3 kinase/AKT signaling pathway, and inhibiting protein synthesis and cell growth [44], was found to be activated in SLFN5 knockdown cells and inhibited by SLFN5 overexpression (Figure 4(a)). Furthermore, pAKT's upstream kinase PI3K is inactivated by PTEN [21, 22], which was found to be downregulated at both the mRNA and the protein level in SLFN5 knockdown cells and enhanced in overexpressing cells (Figures 4(a) and 4(b)). Immunohistochemical staining of SLFN5 and PTEN presented strong positive staining of both proteins in normal lung tissues; however, only weak or negative staining was observed in human lung adenocarcinoma samples (Figure 4(c)). Taken together, these findings demonstrate that SLFN5 promotes PTEN mRNA and protein expression, thereby suppressing PI3K/AKT/mTOR pathways, protein synthesis, and cell proliferation. Meanwhile, SLFN5 suppresses AKT/GSK-3*β*/*β*-catenin, thereby inhibiting proliferation and promoting apoptosis in lung cancer cells.

## 4. Discussion

Lung cancer is a significant threat to human health with high incidence and mortality among malignant tumors. Increasing findings have shown that human SLFN5 functions in malignant tumors, such as melanoma, renal cell carcinoma, and glioblastoma, where it seems to play differential roles, either inhibitory or permissive. We performed lentiviral-mediated stable knockdown and overexpression of the SLFN5 gene in a lung adenocarcinoma cell line to determine the role of human SLFN5 in growth, proliferation, and apoptosis. SLFN5 knockdown promoted lung cancer cell proliferation and growth both *in vitro* and *in vivo*, whereas overexpression of SLFN5 inhibited these processes. SLFN5 knockdown promoted apoptosis, whereas SLFN5 overexpression inhibited it. Mechanistically, SLFN5 plays these antitumor roles through upregulating PTEN, which inactivates PI3K/AKT/mTOR pathways. This is the first report that human SLFN5 exerts inhibitory roles in lung cancer cell tumorigenesis and progression, providing a potential target for future drug development in lung cancer therapy.

Mouse Slfn5 exhibits important antineoplastic effects on mouse renal cell carcinoma cells [11]; however, human SLFN5 did not influence the proliferation of human renal cell carcinoma cells [9]. This does exclude the results of differential experiment methods, since another report of human SLFN5 inhibitory roles in proliferation reported that knockdown of human SLFN5 promoted soft agar colony formation/anchorage-independent growth of human melanoma cells [8]. The inhibitory role of human SLFN5 in melanoma cells is consistent with our present findings in human lung cancer cells. To verify our results, we employed various methods, including counting cell numbers, CCK-8 assay, Ki-67 immunostaining, colony formation, and cyclin D1, and these experiments all yielded consistently supportive evidence that SLFN5 plays inhibitory roles in lung cancer cell proliferation. In addition to these *in vitro* observations, subcutaneous tumor growth in nude mice, an internal microenvironment rich in regulatory factors and surrounding matrices, also supported this conclusion.

Tumor growth depends on both rapid proliferation and antiapoptotic ability. Except for mature blood cells, most normal cells in the human body, such as epithelial and endothelial cells, need to adhere to their surrounding extracellular matrix for survival and normal function and apoptosis occurs once these cells are separated from the extracellular matrix. However, almost all types of cancer cells develop the ability to evade apoptosis. Until now, none of the SLFN family members have been reported to modulate cancer apoptosis. We adopted TUNEL detection and flow cytometry analysis, examining two key apoptosis molecules, Bax and cleaved caspase-3, and our observations at all times indicate that SLFN5 is a proapoptotic factor in lung cancer. Bax, localized on the mitochondrial membrane, releases mitochondrial cytochrome C into the cytosol to trigger caspase-3 cleavage and activation of cleaved caspase-3, which then catalyzes the degradation of many key proteins, resulting in apoptosis. In our present work, both Bax and cleaved caspase-3 were decreased in response to silencing of SLFN5; however, these factors were enhanced after induction of elevated SLFN5, together with TUNEL and flow cytometry results, suggesting that SLFN5 promotes apoptosis in A549 cancer cells. Therefore, SLFN5's inhibition on A549 cell growth is a result of both inhibition of proliferation and promotion of apoptosis.

PTEN is a suppressor gene in lung cancer that is regulated by several transcription factors and methylation modifications [32–37, 45–47]. However, whether other regulators are involved has drawn research attention. In the present study, we found that SLFN5 induced PTEN expression at both the mRNA and the protein level. Consistent with SLFN5 expression in lung cancer samples, PTEN was significantly reduced in cancer compared to adjacent normal tissues. We attempted to determine how SLFN5 regulates PTEN at the transcription level using ChIP with an SLFN5 antibody and sequencing chromatin precipitation, but PTEN's promoter region was not included in the chromatin precipitation by either sequencing analysis or real-time PCR determination (data not shown). These findings indicate that SLFN5's regulation of PTEN transcription occurs via an indirect mechanism. PTEN, a phosphatase, dephosphorylates phosphoinositide, thereby inhibiting AKT phosphorylation and the subsequent phosphorylation cascade that includes mTOR (its phosphorylation promotes protein synthesis via the inactivated eIF4E inhibitor 4e-bp1), GSK-3*β* (its phosphorylation is inactive, resulting in its catalysis of its substrate *β*-catenin to be dephosphorylated and translocate into the nucleus to regulate gene expression of factors, such as cyclin D1, and MT1-MMP as we reported previously), and Bax (its phosphorylation causes degradation through ubiquitination).

## 5. Conclusion

In conclusion, SLFN5 exerts inhibitory roles in lung cancer cell tumorigenesis and progression, providing a potential target for future drug development in lung cancer therapy. To further clarify SLFN5's regulation and function, additional studies investigating some aspects such as regulatory factors, signaling details, and structural mutants of SLFN5 need to be undertaken in the future.

## Figures and Tables

**Figure 1:** The effects of SLFN5 knockdown and overexpression on proliferation of A549 lung cancer cells. (a) Western blot analysis of SLFN5 protein expression in A549 lung cancer cells stably transfected with control shRNA (ShCtrl), SLFN5 shRNA (ShSLFN5), lentiviral vector (Vector), and lentiviral SLFN5 (SLFN5). (b) Immunofluorescence staining of SLFN5 (red) and DAPI (blue) in A549 cells stably transfected with ShCtrl or ShSLFN5. Scale bar, 50 *μ*m. (c) Cell numbers in response to increasing or decreasing levels of SLFN5 (mean ± S.D., *n* ≥ 3). (d) Proliferation by CCK-8 assay in response to increasing or decreasing levels of SLFN5 (mean ± S.D., *n* ≥ 3). (e) Immunofluorescence staining of Ki-67 (red) and DAPI (blue). Percentages of Ki-67-positive cells (mean ± S.D., *n* ≥ 3). Scale bar, 100 *μ*m. (f) Colony formation results (mean ± S.D., *n* ≥ 3). (g) Western blot analysis of cyclin D1 expression with densitometry graphs shown below.

**Figure 2:** Effects of knockdown and overexpression of SLFN5 on apoptosis in A549 lung cancer cells. (a, b) Flow cytometry analysis of apoptotic A549 cells stably transfected with ShCtrl or ShSLFN5 (a) and stably transfected with Vector or SLFN5 (b). Fold change in apoptosis is shown with mean ± S.D., *n* = 3. (c, d) Immunofluorescence staining of TUNEL (red) and DAPI (blue) of apoptotic A549 cells stably transfected with ShCtrl or ShSLFN5 (c) and Vector or SLFN5 (d). TUNEL-positive cell analysis (%) shown as mean ± S.D., *n* ≥ 3. Scale bars, 100 *μ*M. (e, f) Western blot analysis of protein expression of Bax, caspase-3, and cleaved caspase-3.

**Figure 3:** The effect of SLFN5 knockdown or overexpression on A549 cell proliferation in vivo. (a, b) A549 cells stably transfected with ShCtrl or ShSLFN5 were injected into the axilla region of nude mice (2 × 10^6^ cells per mouse, *n* = 9), and tumor volume was measured every 5 days. (c, d) After 40 days, mice were sacrificed, and tumor weight was examined (mean ± S.D., *n* = 9). (e, f) A549 cells stably transfected with Vector or SLFN5 were injected into the axilla region of nude mice (1 × 10^7^ cells per mouse, *n* = 8), and tumor volume was measured every 5 days. (g, h) After 35 days, mice were sacrificed, and tumor weight was examined (mean ± S.D., *n* = 8).

**Figure 4:** SLFN5 regulates p-AKT/GSK-3*β*/*β*-catenin and p-AKT/mTOR pathways via transcriptional regulation of PTEN mRNA. (a) Western blot analysis of protein expression of p-AKT, GSK-3*β*, *β*-catenin, mTOR, and PTEN in A549 cells stably transfected with ShCtrl, ShSLFN5, Vector, or SLFN5. (b) Real-time PCR analysis of PTEN in A549 cells stably transfected with ShCtrl, ShSLFN5, Vector, or SLFN5. (c) Immunohistochemistry and H&E staining of SLFN5 and PTEN in lung cancer samples. Red arrowheads indicate cancer cells, and black arrowheads indicate lymphocytes in the cancer stroma. Scale bars, 100 *μ*M. Positive expression analyses of PTEN and SLFN5 were shown as mean ± S.D.

## Data Availability

The data used to support the findings of this study are available from the corresponding author upon request.

## References

[1] Schwarz D. A., Katayama C. D., Hedrick S. M. (1998). Schlafen, a new family of growth regulatory genes that affect thymocyte development. *Immunity*.

[2] Geserick P., Kaiser F., Klemm U., Kaufmann S. H., Zerrahn J. (2004). Modulation of T cell development and activation by novel members of the Schlafen (SLFN) gene family harbouring an RNA helicase-like motif. *International Immunology*.

[3] Neumann B., Zhao L., Murphy K., Gonda T. J. (2008). Subcellular localization of the Schlafen protein family. *Biochemical and Biophysical Research Communications*.

[4] Bustos O., Naik S., Ayers G. (2009). Evolution of the Schlafen genes, a gene family associated with embryonic lethality, meiotic drive, immune processes and orthopoxvirus virulence. *Gene*.

[5] Puck A., Aigner R., Modak M., Cejka P., Blaas D., Stockl J. (2015). Expression and regulation of Schlafen (SLFN) family members in primary human monocytes, monocyte-derived dendritic cells and T cells. *Results in Immunology*.

[6] Tian L., Song S., Liu X. (2014). Schlafen-11 sensitizes colorectal carcinoma cells to irinotecan. *Anti-Cancer Drugs*.

[7] Kovalenko P. L., Basson M. D. (2014). Schlafen 12 expression modulates prostate cancer cell differentiation. *The Journal of Surgical Research*.

[8] Katsoulidis E., Mavrommatis E., Woodard J. (2010). Role of interferon *α* (IFN*α*)-inducible Schlafen-5 in regulation of anchorage- independent growth and invasion of malignant melanoma cells. *The Journal of Biological Chemistry*.

[9] Sassano A., Mavrommatis E., Arslan A. D. (2015). Human Schlafen 5 (SLFN5) is a regulator of motility and invasiveness of renal cell carcinoma cells. *Molecular and Cellular Biology*.

[10] Li M., Kao E., Gao X. (2012). Codon-usage-based inhibition of HIV protein synthesis by human schlafen 11. *Nature*.

[11] Mavrommatis E., Arslan A. D., Sassano A., Hua Y., Kroczynska B., Platanias L. C. (2013). Expression and regulatory effects of murine Schlafen (Slfn) genes in malignant melanoma and renal cell carcinoma. *The Journal of Biological Chemistry*.

[12] Brady G., Boggan L., Bowie A., O'Neill L. A. (2005). Schlafen-1 causes a cell cycle arrest by inhibiting induction of cyclin D1. *The Journal of Biological Chemistry*.

[13] Arslan A. D., Sassano A., Saleiro D. (2017). Human SLFN5 is a transcriptional co-repressor of STAT1-mediated interferon responses and promotes the malignant phenotype in glioblastoma. *Oncogene*.

[14] Taborelli M., Piselli P., Ettorre G. M. (2019). Survival after the diagnosis of de novo malignancy in liver transplant recipients. *International Journal of Cancer*.

[15] Islami F., Goding Sauer A., Miller K. D. (2018). Proportion and number of cancer cases and deaths attributable to potentially modifiable risk factors in the United States. *CA: A Cancer Journal for Clinicians*.

[16] Wan G., Liu Y., Zhu J. (2019). SLFN5 suppresses cancer cell migration and invasion by inhibiting MT1-MMP expression via AKT/GSK-3 *β*/*β*-catenin pathway. *Cellular Signalling*.

[17] Wan G., Zhu J., Gu X. (2020). Human Schlafen 5 regulates reversible epithelial and mesenchymal transitions in breast cancer by suppression of ZEB1 transcription. *British Journal of Cancer*.

[18] Li J., Yen C., Liaw D. (1997). PTEN, a putative protein tyrosine phosphatase gene mutated in human brain, breast, and prostate cancer. *Science*.

[19] Di Cristofano A., Pandolfi P. P. (2000). The multiple roles of PTEN in tumor suppression. *Cell*.

[20] Myers M. P., Tonks N. K. (1997). PTEN: sometimes taking it off can be better than putting it on. *American Journal of Human Genetics*.

[21] Engelman J. A., Luo J., Cantley L. C. (2006). The evolution of phosphatidylinositol 3-kinases as regulators of growth and metabolism. *Nature Reviews Genetics*.

[22] Vanhaesebroeck B., Guillermet-Guibert J., Graupera M., Bilanges B. (2010). The emerging mechanisms of isoform-specific PI3K signalling. *Nature Reviews Molecular Cell Biology*.

[23] Mackay H. J., Gallinger S., Tsao M. S. (2010). Prognostic value of microsatellite instability (MSI) and PTEN expression in women with endometrial cancer: results from studies of the NCIC Clinical Trials Group (NCIC CTG). *European Journal of Cancer*.

[24] You Y., Geng X., Zhao P. (2007). Evaluation of combination gene therapy with PTEN and antisense hTERT for malignant glioma in vitro and xenografts. *Cellular and Molecular Life Sciences*.

[25] Xu J., Li Z., Wang J., Chen H., Fang J. Y. (2014). Combined PTEN mutation and protein expression associate with overall and disease-free survival of glioblastoma patients. *Translational Oncology*.

[26] Romano C., Schepis C. (2012). PTEN gene: a model for genetic diseases in dermatology. *Scientific World Journal*.

[27] Baig R. M., Mahjabeen I., Sabir M. (2011). Genetic changes in the PTEN gene and their association with breast cancer in Pakistan. *Asian Pacific Journal of Cancer Prevention*.

[28] Patel R., Gao M., Ahmad I. (2013). Sprouty2, PTEN, and PP2A interact to regulate prostate cancer progression. *The Journal of Clinical Investigation*.

[29] Marsit C. J., Zheng S., Aldape K. (2005). PTEN expression in non-small-cell lung cancer: evaluating its relation to tumor characteristics, allelic loss, and epigenetic alteration. *Human Pathology*.

[30] Li D. M., Sun H. (1998). PTEN/MMAC1/TEP1 suppresses the tumorigenicity and induces G1 cell cycle arrest in human glioblastoma cells. *Proceedings of the National Academy of Sciences of the United States of America*.

[31] Stambolic V., MacPherson D., Sas D. (2001). Regulation of PTEN transcription by p53. *Molecular Cell*.

[32] Singh B., Reddy P. G., Goberdhan A. (2002). p53 regulates cell survival by inhibiting PIK3CA in squamous cell carcinomas. *Genes & Development*.

[33] Tang Y. A., Chen C. H., Sun H. S. (2015). Global Oct4 target gene analysis reveals novel downstream PTEN and TNC genes required for drug-resistance and metastasis in lung cancer. *Nucleic Acids Research*.

[34] Hettinger K., Vikhanskaya F., Poh M. K. (2007). c-Jun promotes cellular survival by suppression of PTEN. *Cell Death and Differentiation*.

[35] Vasudevan K. M., Gurumurthy S., Rangnekar V. M. (2004). Suppression of PTEN expression by NF-kappa B prevents apoptosis. *Molecular and Cellular Biology*.

[36] Soria J. C., Lee H. Y., Lee J. I. (2002). Lack of PTEN expression in non-small cell lung cancer could be related to promoter methylation. *Clinical Cancer Research*.

[37] Maeda M., Murakami Y., Watari K., Kuwano M., Izumi H., Ono M. (2015). CpG hypermethylation contributes to decreased expression of PTEN during acquired resistance to gefitinib in human lung cancer cell lines. *Lung Cancer*.

[38] Gu X., Wan G., Yang Y. (2020). SLFN5 influences proliferation and apoptosis by upregulating PTEN transcription via ZEB1 and inhibits the purine metabolic pathway in breast cancer. *American Journal of Cancer Research*.

[39] Gu X., Wan G., Chen N. (2019). DGK*ζ* plays crucial roles in the proliferation and tumorigenicity of human glioblastoma. *International Journal of Biological Sciences*.

[40] Weigel M. T., Dowsett M. (2010). Current and emerging biomarkers in breast cancer: prognosis and prediction. *Endocrine-Related Cancer*.

[41] Musgrove E. A., Caldon C. E., Barraclough J., Stone A., Sutherland R. L. (2011). Cyclin D as a therapeutic target in cancer. *Nature Reviews. Cancer*.

[42] Jurgensmeier J. M., Xie Z., Deveraux Q., Ellerby L., Bredesen D., Reed J. C. (1998). Bax directly induces release of cytochrome c from isolated mitochondria. *Proceedings of the National Academy of Sciences of the United States of America*.

[43] Katsuda K., Kataoka M., Uno F. (2002). Activation of caspase-3 and cleavage of Rb are associated with p16-mediated apoptosis in human non-small cell lung cancer cells. *Oncogene*.

[44] Faried L. S., Faried A., Kanuma T. (2006). Inhibition of the mammalian target of rapamycin (mTOR) by rapamycin increases chemosensitivity of CaSki cells to paclitaxel. *European Journal of Cancer*.

[45] Virolle T., Adamson E. D., Baron V. (2001). The Egr-1 transcription factor directly activates PTEN during irradiation-induced signalling. *Nature Cell Biology*.

[46] Patel L., Pass I., Coxon P., Downes C. P., Smith S. A., Macphee C. H. (2001). Tumor suppressor and anti-inflammatory actions of PPAR*γ* agonists are mediated via upregulation of PTEN. *Current Biology*.

[47] Gericke A., Munson M., Ross A. H. (2006). Regulation of the PTEN phosphatase. *Gene*.

